The article "Involvement of Machine Learning Tools in Healthcare Decision Making" was published in 2021. Journal: J Healthc Eng.

# Involvement of Machine Learning Tools in Healthcare Decision Making

**DOI:** 10.1155/2021/6679512

**Published:** 2021-01-27

**Authors:** Senerath Mudalige Don Alexis Chinthaka Jayatilake, Gamage Upeksha Ganegoda

**Affiliations:** Faculty of Information Technology, University of Moratuwa, Katubedda, Moratuwa, Sri Lanka

## Abstract

In the present day, there are many diseases which need to be identified at their early stages to start relevant treatments. If not, they could be uncurable and deadly. Due to this reason, there is a need of analysing complex medical data, medical reports, and medical images at a lesser time but with greater accuracy. There are even some instances where certain abnormalities cannot be directly recognized by humans. In healthcare for computational decision making, machine learning approaches are being used in these types of situations where a crucial data analysis needs to be performed on medical data to reveal hidden relationships or abnormalities which are not visible to humans. Implementing algorithms to perform such tasks itself is difficult, but what makes it even more challenging is to increase the accuracy of the algorithm while decreasing the required time for the algorithm to execute. In the early days, processing of large amount of medical data was an important task which resulted in machine learning being adapted in the biological domain. Since this happened, the biology and biomedical fields have been reaching higher levels by exploring more knowledge and identifying relationships which were never observed before. Reaching to its peak now the concern is being diverted towards treating patients not only based on the type of disease but also their genetics, which is known as precision medicine. Modifications in machine learning algorithms are being performed and tested daily to improve the performance of the algorithms in analysing and presenting more accurate information. In the healthcare field, starting from information extraction from medical documents until the prediction or diagnosis of a disease, machine learning has been involved. Medical imaging is a section that was greatly improved with the integration of machine learning algorithms to the field of computational biology. Nowadays, many disease diagnoses are being performed by medical image processing using machine learning algorithms. In addition, patient care, resource allocation, and research on treatments for various diseases are also being performed using machine learning-based computational decision making. Throughout this paper, various machine learning algorithms and approaches that are being used for decision making in the healthcare sector will be discussed along with the involvement of machine learning in healthcare applications in the current context. With the explored knowledge, it was evident that neural network-based deep learning methods have performed extremely well in the field of computational biology with the support of the high processing power of modern sophisticated computers and are being extensively applied because of their high predicting accuracy and reliability. When giving concern towards the big picture by combining the observations, it is noticeable that computational biology and biomedicine-based decision making in healthcare have now become dependent on machine learning algorithms, and thus they cannot be separated from the field of artificial intelligence.

The article "Involvement of Machine Learning Tools in Healthcare Decision Making" was published in 2021. Journal: J Healthc Eng.

## 1. Introduction

Artificial Intelligence includes approaches and techniques like machine learning, machine reasoning, and robotics. In this review, the main concern will be given towards machine learning as it is the approach that is being applied using different techniques and algorithms in various healthcare activities. The use of machine learning to solve clinical problems is called revolutionary clinical decision making. When machine learning is being used in clinical decision making, it implies that the system will perceive a given individual by collecting and interpreting data relevant for the health of that individual and it will reason on the data to suggest the best actions that need to be performed to maintain or improve the individual's health. In machine learning, the system needs to learn the context of the problem and the quality of data provided. Normally, these algorithms are not very strong and concrete at the beginning, but by performing a single and repetitive task, the algorithm becomes strong with increased number of previous experiences.

There are two distinct ways that a clinical decision-making solution interprets by comparing previous knowledge that is included in the dataset. One is the fast or intuitive approach which uses underlying clinical pattern recognition and is typically used in medical emergencies. But these have a higher possibility of being erroneous and provide incomplete perception. The other approach is the slow or reasoned method. It is deductive, deliberate, and needs greater intellectual, time, and cost information. But the decisions made are more accurate. As all these decisions are based on the data that are being collected, analysed, and stored in complex and heterogeneous forms, it is important to use algorithmic approaches to minimize the computing power required. Machine learning applications have currently contributed massively to the healthcare sector worldwide to improve its quality and will continue to do so [1].

The article "Involvement of Machine Learning Tools in Healthcare Decision Making" was published in 2021. Journal: J Healthc Eng.

It is also important to mention that when discussing computational decision making in the healthcare sector, it is not always about detecting or predicting diseases, biomedicine, biomedical image analysis, etc., but also about how to perform medical treatment research, patient care, allocating resources, managing hospital volume, public health policymaking, and much more. As an example, when considering the current situation that has arisen with COVID-19 pandemic, it could be seen that all the aforementioned points need to be considered in healthcare and those tasks need to be performed within a considerably small time period. Therefore, the best approach is to use machine learning-based decision making in the healthcare sector in such times. This is the reason why there is a demand for the area “emergency machine learning” in the present world [2].

Even though artificial intelligence is set to make transformation by playing an important role in healthcare, there are a few ethical aspects as well that need to be considered when implementing such systems and obtaining decisions from them. Few of the ethical issues are the accountability and transparency of the decisions made by such systems, the potential for group harms arising from algorithmic bias and the professional roles, and the integrity of the clinicians. Therefore, it is important to give consideration when implementing such systems and balance them with the benefit that they create with more efficient healthcare systems by the high and accurate computational power of artificial intelligence at a considerably low cost. Moreover, algorithms in artificial intelligence have the capacity to perform computerized predictive analysis by filtering, ordering, and searching for patterns from big datasets from multiple sources to provide fast and informed decisions. In the present context, due to this discussed matter, most jurisdictions do not allow directly applying these algorithms to make the final decisions, but instead use them as an aid for diagnosis [3].

Throughout the paper many machine learning algorithms and their applications in the field of computational decision making for healthcare will be discussed along with the methods that are used to improve the efficiency of the algorithms with the objective to highlight the importance of scalable machine learning algorithms in healthcare applications. The aim of the paper is to discuss the involvement of machine learning algorithms in the healthcare sector to perform computational decision making starting from the initial phase where machine learning was introduced to computational biology till the peak it currently stands which is the introduction of precision medicine to the field of biomedicine. This paper is organized in different sections. Machine learning approaches and algorithms that are being applied in healthcare for decision making will be discussed in Section 2 followed by the applications of machine learning in the healthcare sector in various aspects such as disease prediction and detection, medical imaging, machine learning in biomedicine, biomedical event extraction, machine learning approaches to polypharmacology, and machine learning for drug repurposing using system biology. The discussion section will include an evaluation and comparison of machine learning algorithms with regard to the applications of these algorithms in healthcare which will be followed by recognition of different mechanisms used to enhance the accuracy of the algorithms within applications, along with further information on the involvement of scalable machine learning algorithms for computational decision making in healthcare. The latter part of the paper consists of the conclusion.

The article "Involvement of Machine Learning Tools in Healthcare Decision Making" was published in 2021. Journal: J Healthc Eng.

## 2. Machine Learning Approaches and Algorithms

Machine learning can be introduced as a scientific discipline that focuses on how computers learn from data and continuously improve themselves. It is mainly based on probability and statistics. But it is more powerful than the standard statistical methodologies when it comes to decision making. Information gathered from a dataset which is being given to the algorithm is called features. The accuracy of the predictions made by the model is dependent on the quality of the features provided to the algorithm. It is the duty of a machine learning developer to detect the subset of features that could best fit the purpose, increasing the accuracy of the model. This is not an easy task. Continuous experiments should be carried out to identify the said feature subset for the algorithm. When considering putting a machine learning algorithm to applications, there are basically three steps to follow, which are training, testing, and validation. Training is important as the accuracy of the results will be depending on the training dataset. Using the test dataset, the performance of the algorithm will be measured. When using the test data for measuring the performance, it is also important to lower the bias and to increase the variance in this testing period. A good machine learning algorithm must optimize the bias-variance trade-off. The evaluation of the final machine learning algorithm performance is done based on the validation dataset in the validation period [4]. As a start, it would be better to have an idea about various approaches taken in machine learning along with several algorithms that are being used excessively for clustering and classification purposes in machine learning.

The article "Involvement of Machine Learning Tools in Healthcare Decision Making" was published in 2021. Journal: J Healthc Eng.

### 2.1. Supervised Learning

In supervised learning, a training set is provided with appropriate objectives in this approach. Classification and regression are the two categories found in supervised learning. In classification, with the use of classification methods, the trained system allocates inputs into classes. In regression, the sources are continuous rather than discrete. The root-mean-squared error is being used to evaluate regression predictions, while accuracy is being used to evaluate classification predictions. [5]. Supervised learning has the goal of predicting a known output based on a common dataset. Tasks performed by supervised learning can most of the time be performed by a trained person as well. Supervised learning focuses on classification which involves choosing among subgroups to best describe a new instance of data and prediction, which involves estimating an unknown parameter. This is often used to estimate and model risk while finding relationships which are not readily visible to humans [6]. Below are a few supervised learning algorithms which are widely used in the field of computational biology and biomedicine.

#### 2.1.1. K-Nearest Neighbour (KNN)

KNN is a popular supervised classification algorithm which is used in many fields such as pattern recognition, intrusion detection, and so on. KNN is a simple algorithm which is easy to understand. Even the accuracy is high in KNN, but the issues are that it is computationally expensive and it has a high memory requirement as both testing and training data need to be stored [7]. A prediction for a new instance is obtained by finding the most similar instances at first and then summarizing the output variable according to those similar instances. For regression, this can be the mean value, and for classification, this may be the mode value. To determine the similar instance, the distance measure is used. Euclidean distance is the most popular approach used to calculate the distance. The training dataset should be vectors in a multidimensional feature space, each with a class label [5].

#### 2.1.2. Support Vector Machine (SVM)

SVM is a supervised machine learning algorithm which is used to address mainly classification problems but also used for regression issues. In this algorithm, initially, the data items are plotted as points in an n-dimensional space with the feature value being the particular coordinate. Then, it identifies the hyperplane that separates the datapoints into two classes. By this, the marginal distance between the decision hyperplane and instances that are close to the boundary can be maximized [5].What brings SVM ahead of other algorithms is that it has basic functions that can map points to other dimensions by using nonlinear relationships [8]. As it divides the datapoints to two classes, SVM is also known as the nonprobabilistic binary classifier. SVM has more accuracy when compared with many other algorithms. But it is best suited for problems with small datasets. The reason is that when the dataset keeps on getting larger, the training becomes more complex and time consuming. When data have noise, it cannot perform well. To make the classification more efficient, SVM uses a subset of training points. SVM is capable of solving both linear and nonlinear problems, but nonlinear SVM is preferred over linear SVM as it has better performance [7].

The article "Involvement of Machine Learning Tools in Healthcare Decision Making" was published in 2021. Journal: J Healthc Eng.

#### 2.1.3. Decision Trees (DTs)

DT is a supervised algorithm which has a tree like model where decisions, possible consequences, and their outcomes are being considered. Each node carries a question, and each branch represents an outcome. The leaf nodes are class labels. When a leaf node is being reached by a sample data, the label of the corresponding node will be assigned to the sample. This approach is suited when the problem is simple and when the dataset is small. Even though the algorithm is easy to understand, it has certain issues such as the overfitting problem and biased outcomes when working with imbalanced datasets. But DT is capable of mapping both linear and nonlinear relationships [7].

#### 2.1.4. Classification and Regression Trees (CARTs)

CART is a predictive model from which the output value is predicted based on the existing values in the constructed tree. The representation for the CART model is a binary tree in which each root represents a single input and a split point on that variable. Leaf nodes contain an output which is used to make predictions [5].

#### 2.1.5. Logistic Regression (LR)

LR is a popular mathematical modelling procedure which is used for epidemiologic datasets in the area of machine learning. It first calculates using the logistic function. Then, it learns the coefficients for the logistic regression model and then finally makes predictions using that logistic regression model [9]. This model is a generalized linear model and has two parts, namely, linear part and link function. The linear part is responsible for carrying out the calculations of the classification model, and the link function is responsible for delivering the output of the calculation [10]. LR is a supervised machine learning algorithm which needs a hypothesis and a cost function. It is to be noted that optimizing the cost function is important [11].

The article "Involvement of Machine Learning Tools in Healthcare Decision Making" was published in 2021. Journal: J Healthc Eng.

#### 2.1.6. Random Forest Algorithm (RFA)

RFA is a trending machine learning technique which is capable of both regression and classification [12]. It is a supervised learning algorithm in which the ground methodology is recursion. In this algorithm, a group of decision trees are being created and the bagging method is used for training purposes [13]. RFA is insensitive to noise and can be used for imbalanced datasets. The problem of overfitting is also not prominent in RFA [7].

#### 2.1.7. Naive Bayes (NB)

NB is a classification algorithm which is used for binary and multiclass problems. The NB classifiers are a collection of classifying algorithms that are based on the Bayes theorem. But they all adhere to a common principle which is every pair of features being classified must be independent of each other [5]. This is a bit similar to SVM, but the process takes advantage from statistical methods. In this method, when there is a new input, the probabilistic value will be calculated among the classes with regard to the given input and the data will be labelled with the class which has the highest probabilistic value for the given input [9].

#### 2.1.8. Artificial Neural Network (ANN)

ANN is a supervised machine learning approach which is well known for image classification problems. In machine learning, artificial neurons are considered to be the basic concept of ANN and it is similar to a biological neural network. There are 3 layers in an ANN, and every node in each layer is connected with all the nodes in the other layers. By increasing the number of hidden layers, a deeper neural network can be created [14]. In neural networks, there are three types of functions. Error function will determine how good or bad the output was for a given set of inputs. The search function will identify the changes that would reduce the error function. Update function will determine how the changes will be made as per the search function. This is an iterative process that would improve the performance of the algorithm [8].

### 2.2. Unsupervised Learning

When a developer does not have a clear understanding of the data that are involved with the system, it is not possible to label the data and provide them as the training dataset. In these cases, the machine learning algorithms themselves can be used to detect similarities and differences between the data objects. This is the unsupervised approach of machine learning. In this method, existing patterns will be identified and the data will be clustered according to the identified patterns [4]. Therefore, in unsupervised learning, the system makes decisions without being trained by a dataset as no labelled data are being given to the system which could be used for predictions [5]. It is to be noted that unsupervised learning is an attempt to find naturally occurring patterns or groups within data. The challenging part in it is to find whether the recognized patterns or groups are useful in some way. This is the reason for unsupervised learning to play a major role in precision medicine. As a simple example, when grouping individuals according to their genetics, environment, and medical history, certain relationships among them which were not visible before might get identified by unsupervised machine learning algorithms [6]. K-means, mean shift, affinity propagation, density-based spatial clustering of applications with noise (DBSCAN), Gaussian mixture modelling, Markov random fields, iterative self-organizing data (ISODATA), and fuzzy C-means systems are a few examples for unsupervised algorithms [8].

The article "Involvement of Machine Learning Tools in Healthcare Decision Making" was published in 2021. Journal: J Healthc Eng.

Clustering is an approach in unsupervised learning, and it can be used for dividing inputs into clusters. But these clusters are not identified initially but are grouped based on resemblance [5]. In clustering, the root approaches are separated as per the different features that they carry. They can be partitioning (k-means), hierarchical, grid-based, density-based, or model-based, and they can be further divided as numerical, discrete, and mixed data types. Inheritance relationships between clustering algorithms within an approach show common features and improvements that they make on each other. Speed, minimal parameters, robustness to noise, outliers, redundancy handling, and object order independence are the desired clustering features which are required in a clustering algorithm to be implemented within a biomedical application [15]. Clustering algorithms are used when datasets are too large and complex for manual analysis. Therefore, they must be fast and they must not be affected by redundant sequences. It is important to evaluate a clustering algorithm to know whether it is suitable for the problem in hand by considering features such as

1. Scalability: runtime and memory requirements should not exceed when working with large datasets.
2. Robustness: ability to detect outliers that are different from the rest of the samples.
3. Order insensitivity: the order that the inputs are given should not be affecting the final output.
4. Minimum user-specified input: the minimum number of parameters that should be provided.
5. Mixed data types: the objects provided may have different data types.
6. Arbitrary-shaped cluster: ability to find arbitrary-shaped clusters.
7. Point proportion admissibility: duplicating objects and reclustering should not change the result [15].

The article "Involvement of Machine Learning Tools in Healthcare Decision Making" was published in 2021. Journal: J Healthc Eng.

When giving concern to the above factors, it is to be noted that as a result of the use of unsupervised machine learning in healthcare, when a patient is being diagnosed for a specific disease, in that process itself the patient will be identified of another disease as well if any such disease is present. The reason is that the algorithm has learnt itself on facts that need to be considered for various types of diseases and it analyses the given data and categorizes as diseases according to those data. In addition, even though various reports taken to identify diseases may include different types of data, using this approach, all these data can be analysed simultaneously which is of much convenience and also time saving. With regard to the aforementioned aspects, there is no doubt that healthcare decision making is highly benefited from the unsupervised machine learning approach.

#### 2.2.1. Partition Clustering

In partition clustering, the objects are partitioned and may change clusters based on the dissimilarity. It is useful in bioinformatics when the number of clusters is decided such as for a small gene expression dataset. The drawback is that the user needs to manually enter the number of clusters as an input. But this approach is commonly used in bioinformatics. Fuzzy k-means, COOLCAT, clustering large applications (CLARA), and clustering large applications based on randomized search (CLARANS) are a few examples for partition clustering algorithms [15].

#### 2.2.2. Graph-Based Clustering

Graph-based clustering is used in interactomes to make complex predictions and to sequence networks. This approach is often slow and sensitive to user-specified parameters. super-paramagnetic clustering (SPC), Markov cluster algorithm (MCL), molecular complex detection (MCODE), and restricted neighbourhood search cluster (RNSC) are a few examples for graph-based clustering algorithms [15].

#### 2.2.3. Hierarchical Clustering

In hierarchical clustering, the objects are partitioned into a tree of nodes and these nodes are considered as clusters. There are parent nodes and child nodes. A node could have just one parent, and each node can have zero or more child nodes. This approach is popular in bioinformatics as clusters can be navigated at various levels of granularity. The drawbacks are that they are often slow, errors made when merging clusters cannot be undone even though it affects the result, and if large clusters are merged, then interesting local cluster structure may be lost. This approach is used to represent protein sequence family relationships and also could be used to show gene relations reflecting their gene similarity. Chameleon, robust clustering using links (ROCK), scalable information bottleneck (LIMBO), and spectral are a few examples for hierarchical clustering algorithms [15].

The article "Involvement of Machine Learning Tools in Healthcare Decision Making" was published in 2021. Journal: J Healthc Eng.

#### 2.2.4. Density-Based Clustering

Density-based clustering uses a local density criterion, and the clusters are subspaces in which the objects are dense and are separated by subspaces of low density. It is used in bioinformatics to find the densest subspaces in interactome networks, typically involving cliques. Time efficiency and the ability to find clusters of arbitrary shapes are the advantages of this approach. Some of these algorithms accept user parameters, but it is not the number of clusters. Ordering points to identify the clustering structure (OPTICS), clustering in quest (CLIQUE), density based clustering (DENCLUE), and clustering categorical data using summaries (CACTUS) are a few examples for density-based clustering algorithms [15].

#### 2.2.5. Model-Based Clustering

In model-based clustering, it is assumed that objects match a model which is often a statistical distribution. The model can be user specified using a parameter, and this model can even be changed in the process. This approach can be found in bioinformatics to integrate background knowledge into gene expressions, interactomes, and sequences. Slow processing time on large datasets is a drawback of this method. If the user assumptions are false when defining the models, then the results will also be inaccurate. SVM-based clustering, COBWEB, and AutoClass are a few model-based clustering algorithms [15].

### 2.3. Semisupervised Learning

For semisupervised learning, a partial training set of data is provided. This type of training is used when some missing results could be targeted by some training data. Semisupervised learning algorithms are trained on both labelled and unlabelled data. Due to this reason, it exhibits the features of both supervised and unsupervised machine learning algorithms [16].

### 2.4. Evolutionary Learning

Evolutionary learning is mainly used in the biology field to learn about biological organisms and predict their survival rate. Using this method, the level of correctness of a result can also be predicted [16].

### 2.5. Active Learning

In active learning, the system gets the training tags only for a restricted set of occurrences. By using it, the optimality of the substances can be enhanced to gain tags for the required goal. The advantage in this approach is that the algorithm not only continuously learns but also gets the facts which were self-learnt approved either by querying a user or an information source in an interactive manner. It is something similar to budget functions in an organization and is a modern machine learning approach for decision making [16].

The article "Involvement of Machine Learning Tools in Healthcare Decision Making" was published in 2021. Journal: J Healthc Eng.

### 2.6. Deep Learning

Deep learning is an advanced phase of machine learning which evolves around neural networks for learning and predicting data. Using this approach, complex generalized systems can be implemented which are able to accept any type of problem and give predictions regarding it [16].

### 2.7. Reinforcement Learning

In reinforcement learning, the training data are provided only as a response to the program's activities in a self-motivated situation. It has a continuous learning process from the environment in an iterative fashion [13].

After discussing several machine learning approaches, it would be better to list down a few examples on the applications of machine learning in the field of biomedicine so that this review will be interesting from the very beginning. In neuroscience, machine learning classifiers are being used to study functional and structural dynamics of the brain. Machine learning approaches are used in cancer prediction and prognosis. SVM classifiers are used to detect prostate cancer. Hierarchical clustering has been used in investigation of Alzheimer's disease. ANN has been used in classifying different subtypes of psychogenic nonepileptic seizures [4]. With the knowledge gathered on various machine learning approaches and machine learning algorithms which are mostly connected with computational biology and biomedicine, now it is time to dive into deeper knowledge and to identify the applications of these algorithms in the discussing field.

## 3. Machine Learning in Disease Prediction and Detection

Various machine learning approaches have been implemented to predict or detect a disease at its early stages so that the treatment for it would be less complex and it would increase the probability of the patient being cured. As a result of these approaches, different types of diseases have been detected but with diverse accuracy levels depending on factors such as the used algorithm, feature set, training dataset, and so on. In this section, a few selected diseases will be discussed as examples, along with the importance of identifying a disease at the earliest, the machine learning methods implemented to detect the disease, and the features that were considered to make predictions. A descriptive comparison of the machine learning approaches which have been implemented will be conducted in the discussion section of the paper, followed by suggestions to further improve them.

### 3.1. Cancer

Human body has the right count of cells of each type. Cancer begins with abrupt changes in the cell organization. Signals which are being generated by cells determine the control and division of cells. When these signals become faulty, cells multiply too much which form a lump called tumour. Nowadays, thermography is more reliable as it is noninvasive and nonionizing. With the emerging technology, it has been producing efficient and positive results which have made it superior over other technologies. From the thermographic images, with the use of feature extraction techniques and machine learning techniques, the presence of cancer cells can be detected. Scale invariant feature transform (SIFT) and speeded up robust feature (SURF) techniques can be used to extract features from images. Using principal component analysis (PCA), the features could be further filtered in order to make better interpretations [7].

The article "Involvement of Machine Learning Tools in Healthcare Decision Making" was published in 2021. Journal: J Healthc Eng.

#### 3.1.1. Breast Cancer

Breast cancer is a type of cancer that is mostly seen in women and is a leading cause for women's death. But this can be reduced by early detection of cancerous cells by tests like magnetic resonance imaging (MRI), mammogram, ultrasound, and biopsy. Breast cancer is diagnosed by classifying the tumour. Tumours can be either benign or malignant. It is to be noted that malignant tumours are more harmful than benign tumours. But it is not an easy task for physicians to distinguish among these tumours. This makes machine learning algorithms important as they can automatically learn and improve from the experiences without being explicitly programmed [5].

In the past years, many machine learning techniques were developed for breast cancer detection and classification. Their process could be analysed in three stages which are preprocessing, feature extraction, and classification. Feature extraction stage is important as it helps in discriminating between benign and malignant tumours. Then, the image properties such as smoothness, coarseness, depth, and regularity are extracted using segmentation [17].

Normally, images are converted to binary to extract useful information. But it has been observed that once doing so, some important features in the image vanished which omits crucial information. This has led to keeping the images in the grey scale format. Using discrete wavelet transformation (DWT), the images can be transformed from the time domain to the frequency domain. This wavelet decomposition contains four matrices which are the approximation coefficient matrix, the horizontal detailed coefficient matrix, the vertical detailed coefficient matrix, and the diagonal detailed coefficient matrix. These are the values that will be used for the machine learning algorithms [11].

#### 3.1.2. Lung Cancer

Lung cancer can initiate in the windpipe, main airway, or lungs. People with emphysema and previous chest problems have a higher probability of being diagnosed with lung cancer. Tobacco, smoking, and air pollution can be a few major risk factors for lung cancer. Lung cancer starts in the lungs at the primary stage and spreads to other organs as the secondary stage. Symptoms of lung cancer will not be shown until the disease is quite advanced. That is what makes it more dangerous [9].

The article "Involvement of Machine Learning Tools in Healthcare Decision Making" was published in 2021. Journal: J Healthc Eng.

Computerized tomography (CT) reports are less noisy as compared to MRI and X-ray reports. Grayscale conversion, noise reduction, binarization, and segmentation techniques are important to get the image in the required form with less noise and distortion. When converting to grey scale, the average of RGB is taken. The median filter is used for noise reduction. Segmentation removes unnecessary details from the images and locates the objects and the boundaries. In feature extraction stage, features such as area, perimeter, and eccentricity are considered [18].

Small-cell lung cancer (SCLC) detection is extremely difficult for human as it is almost identical to the one without. This is where the machine learning algorithms such as convolution neural network- (CNN-) based deep learning methods could be used in detecting SCLC. Usually, deep learning algorithms require large training datasets which is an issue. Entropy degradation method (EDM) can be used to overcome the said matter. The training data and testing data need to be high-resolution lung CT scans. EDM carries the concept of shallow neural network where vectorized histograms are converted to scores. Then, the scores are transformed to probability using logistic function. In this approach, SCLC detection is considered as a binomial problem which contains only two groups: either a healthy person or a lung cancer patient. So, initially test data are also given with both these types. This approach is reasonably accurate but not the best, and there is a large space to be further improved. But it is recommended that it could be further improved by providing a larger training set and a deeper network. By combining with CNN, the image processing is also further improved for better detection as CNN is being used in many applications of CT imaging [19].

#### 3.1.3. Acute Lymphoblastic Leukaemia

Acute lymphoblastic leukaemia (ALL) is a type of cancer where a large number of immature lymphocyte blood cells develop and they affect the production of other blood cells. This progresses rapidly and can be very fatal within a month or a week. Pale colour of skin, patient feeling very tired, lymph node getting enlarged, fever, and joint pain are a few symptoms that were identified in the patients who were diagnosed with ALL. Machine learning algorithms play a vital role when trying to automatically segment and classify microscopic images to detect leukaemia.

The article "Involvement of Machine Learning Tools in Healthcare Decision Making" was published in 2021. Journal: J Healthc Eng.

There have been various machine learning algorithms used for leukaemia detection such as KNN, SVM, NB, radial basis function network (RBFN), and multilayer perceptron (MLP). But in all these approaches, there are basically four sections which are preprocessing, feature extraction, classification model building, and evaluation of the classifier. In the preprocessing stage, cropping of the image will be done so that the region of interest (ROI) is clearly visible and the unwanted information is eliminated. Using the Gaussian blur smoothing technique, the images can be further processed to enhance the picture by reducing the noise. In the feature extraction stage, concern is given towards colour-based features, geometrical features, statistical features, Haralick texture feature, image moments, local binary pattern, and presence of adjacent cells [20].

### 3.2. Diabetes

Diabetes is a chronic disease, and it needs to be identified at the early stages for correct medication. Diabetes is caused when the sugar ratio in blood increases. This makes the life complicated for the patients due to many reasons. Diabetes can be classified under three types, namely, diabetes 1, diabetes 2, and gestation diabetes.

Discriminant analysis (DA) is a procedure in which the class label of an input is determined by a series of equations that are obtained by input features. Normally, DA uses two possible objectives which are finding a related equation for classifying test samples and interpretation of the predictive equation to better understand the relationship among features. Being pregnant, the weight of the patient, blood pressure, glucose concentration, the ratio of insulin in blood, diabetes pedigree function (DPF), skinfold thickness, and patient age are some features which can be considered for the classification [10].

By using machine learning algorithms such as Gaussian Naive Bayes (GNB), LR, KNN, CART, RFA, and SVM along with variables in electronic medical records (EMRs) such as serum-glucose1, serum-glucose2 levels, body mass index (BMI), age, race, gender, creatinine level, and so on, prediction of type 2 diabetics was possible [21]. Time to time various machine learning techniques were used to try and improve the accuracy of the predictions made. One approach was made using neural networks. In this method, a feed-forward neural network was trained by a backpropagation algorithm. Even in this approach, the features that were considered are the number of pregnancies, skinfold thickness, serum-insulin, BMI, DPF, and age and the main feature considered was the plasma-glucose level. It was observed that the predictions made by using neural networks showed a higher accuracy, when compared with other machine learning algorithms [22]. Research has been carried out on using deep neural networks (DNNs) as well for prediction of diabetics by training the DNN using five-fold and ten-fold cross validation. It is to be highlighted that both aforementioned approaches which were taken using neural networks have shown an accuracy near 97% in diabetes prediction [23].

The article "Involvement of Machine Learning Tools in Healthcare Decision Making" was published in 2021. Journal: J Healthc Eng.

### 3.3. Heart Diseases

Heart diseases are severe events which are caused by blockage inside the heart arteries. Chronic heart disease is the rise of plaque inside the coronary arteries. This progresses slowly and could lead to a heart attack. Peculiar glucose metabolism, extreme blood pressure, dyslipidaemia, smoking, lack of physical exercise, and age are few risk factors that have been identified for major heart diseases. Symptoms of a heart disease may include shortness of breath, weakness of physical body, swollen feet and fatigue with related signs, and so on [14].

In the field of cardiology, the tasks that precision medicine has performed include diagnostics as well as therapeutics in various subfields. Interventional cardiology, personalized treatment options in correcting heart rhythms, some gender differences affecting the outcome of cardiovascular diseases, and numerous works done in genomics can be highlighted as areas in which tasks have been performed by precision medicine in cardiology. Nowadays, in healthcare informatics, there are services such as patient monitoring and clinical decision support systems (CDSSs). With the advancement of machine learning, now complex problems can be solved even by machines which was only possible by humans, decades back. By utilizing these techniques in precision medicine, the CDSS could be modified to make complex clinical decisions, recognizing newer phenotypes and planning person-oriented specialized treatment options.

In cardiology, blood tests are popular among the different investigation methods in precision medicine. AGES is a specific precision medicine test which utilizes other factors in addition to blood tests to avoid ischemic heart disease. In precision medicine, concern is mainly given towards genetics and there are many research studies being carried out to find genetic causes of a disease. Cardiac genetics, cardiac oncology, and ischemic heart disease can be identified as specific areas of interest in precision cardiology. Methods such as blood tests, genetics tests, image tests, or even a combination of them may be used for diagnostic and therapeutic purposes when advancing with precision medicine in cardiology. Many cardiovascular diseases have their roots embedded in genetics. Therefore, solutions using precision medicine are considered more productive specially in these types of diseases. CNN, recurrent neural network (RNN), natural language processing (NLP), SVM, and long short-term memory (LSTM) are few machine learning techniques which could be used efficiently to make precise CDSS using deep learning [24].

The article "Involvement of Machine Learning Tools in Healthcare Decision Making" was published in 2021. Journal: J Healthc Eng.

A machine learning approach to identify cardiologic diseases includes preprocessing, feature selection, cross validation method, machine learning classifiers, and classifier performance evaluation. There are several preprocessing techniques such as removing of missing values, standard scalar, and MinMax scalar. Feature selection is important in machine learning as irrelevant features can affect the classification performance of the algorithm. By applying feature selection prior to the classification, the execution time is reduced and the accuracy of the classification is increased. There are various feature selection algorithms. Relief, Minimal Redundancy Maximal Relevance (mRMR), and Least Absolute Shrinkage and Selection Operator (LASSO) are a few popular feature selection algorithms [25].

### 3.4. Chronic Kidney Disease (CKD)

CKD is a type of a kidney disease which gradually affects the kidney functionality and leads to kidney failure. CDK can be diagnosed using clinical data, lab tests, imaging studies, and biopsy. But biopsy has some disadvantages such as being invasive, costly, time-consuming, and sometimes being risky. This is where machine learning can be applied to overcome the aforementioned disadvantages. In many disease predictions using machine learning, SVM was a commonly used classifier. But for CKD, there is not much research that could be found that uses SVM for the classification. ANN, DT, and LR were the main machine learning classifiers used in this domain. When observing the obtained results, ANN showed far better performance when compared with DT and LR on CKD diagnosis [26].

### 3.5. Parkinson's Disease (PD)

PD is a chronic and progressive movement disorder. It has no causes, no permanent cure, and limited treatment options. It is found that PD occurs due to reduced production of dopamine, a chemical that controls movement and coordination. Tremors, rigidity, slowness of movement, and postural instability are a few symptoms of PD. Abnormal writhing movement is a significant symptom of this disease. Some researchers have applied machine learning algorithms on video recordings and computer vision to differentiate healthy controls from PD patients. Some researchers have also used voice samples to differentiate healthy controls from PD patients [27]. PD belongs to the neurodegenerative disease category that may directly or indirectly affect the brain cells which will result in affecting movement, speech, and other cognitive parts [28].

The article "Involvement of Machine Learning Tools in Healthcare Decision Making" was published in 2021. Journal: J Healthc Eng.

The feature set for the classification can be obtained based on PCA and genetic algorithm (GA). GA is inspired by Darwin's theory of evolution. A variable is considered as a gene. Chromosomes are a sequence of a gene. A predefined function evaluates the quality of a chromosome and the high-performing chromosome will be used to create the offspring. Genetic operations such as mutation and crossover are used to create the offspring. Basically, it is a competition between the chromosomes in which the fittest will survive till the end. This is the concept which will be behind the feature extraction using the GA [29]. PCA is an unsupervised linear conversion technique and a statistical technique commonly used to identify new patterns in high-dimensional data. Common applications that use PCA are face recognition and image compression [30].

### 3.6. Dermatological Diseases

Dermatological diseases are complex and have a large variety, and people have scarce expertise on it. Early detection is always preferred as it could lead to serious outcomes. Eczema, herpes, melanoma, and psoriasis are a few dermatological diseases which should be identified at the early stage to take life out of danger.

In one approach that was taken to diagnose dermatological diseases, the first phase involved data collection and data augmentation using images. Phase 2 is very important as it is where the model is created and trained. In the last phase, the image is converted to an array and the features are broken down using the trained model that was created. There are various augmentation techniques such as synthetic minority oversampling technique (SMOTE) and computer vision techniques like grey scaling, blurring, increasing contrast, changing the colour channel, sharpening, reducing the noise, and smoothing. When there are more instances in the database, it is better for the training of the model. Training the CNN with a large dataset overcomes the overfitting problem. SVM classifier is used for the prediction. The features in the final convolutional layer can be directly given to the SVM as an input. But in order to do this, the SVM must be trained by giving the trained features from the final convolutional layer as the training dataset. Then, the SVM will convert it to vectors and store them [31].

## 4. Machine Learning in Medical Imaging

Medical imaging is a rapidly growing research area as it is important to diagnose diseases in many instances. Several steps can be identified when observing the process of making predictions from an image using machine learning. Once an image is given as the input, it will be divided into different segments to zoom the interested area. Then, with the use of information retrieval techniques, features can be extracted from those areas. Among them, the required features are selected and the noise is removed. Finally, the classifier will classify the extracted data and will make predictions based on the classification.

The article "Involvement of Machine Learning Tools in Healthcare Decision Making" was published in 2021. Journal: J Healthc Eng.

Nowadays, in the medical community, accurate diagnosis of a disease by processing large amounts of medical data is crucial. In the field of medicine and biology, there are various tasks which are being carried out using machine learning algorithms. Distribution of data on the basis of their characteristics, medical data examination, disease diagnosis and treatment planning, data gathering and inspection, correcting diagnostic of different diseases by medical imaging, and extracting features from medical images on diseases are just a few of the applications.

When further consideration is given towards the applications of medical imaging, it can be observed that medical imaging is extensively being used to improve planning of surgical procedures with regard to many diseases. Therefore, before discussing the involvement of machine learning in medical imaging, below mentioned are a few such applications that would better explain how medical imaging is being applied in surgical planning to obtain positive results while mitigating the risks.

As the skull is one of the most complex areas in a human body in both anatomical and surgical perspectives, surgical management is extremely difficult when working with a wide variety of lesions. But during the last decades, the endonasal endoscopic route was considered as a suitable approach for several skull-based lesions. A main advantage is that when performing a skull-based surgery through the nose with the aid of an endoscope, direct visualization of neurovascular structures of different areas of the skull base can be obtained with minimum brain displacement and manipulation. The endoscope also provides a wider and multiangle close-up view which is of much importance in the surgical field [32]. For diseases like rectal cancer, MRI plays a key role as it can accurately depict the local extent of the cancer and generates relevant information required for prognoses which can directly influence the choice of the optimal therapeutic procedure used for each individual patient which encourages the area of personalized medicine [33].

The article "Involvement of Machine Learning Tools in Healthcare Decision Making" was published in 2021. Journal: J Healthc Eng.

It is to be noted that when image-guided surgeries are compared with conventional surgical approaches, image-guided surgeries are less invasive, have more precise targeting, and have improved outcomes. Imaging is used to plan, monitor progress, and to assess results. In neurosurgery, this is more crucial as the object of the surgical procedure is hard to be located and needs to be reached with minimum damage to the healthy tissues. Apart from it, to guide the placement of the surgical instruments and to ensure that the required tissue is being treated, medical imaging is vital. At present, a wide variety of medical imaging modalities are being used such as magnetic resonance imaging, computed tomography, ultrasound, positron emission tomography, single-photon emission computed tomography, fluoroscopy, and so on to perform different assessments like biopsies, tumour resection, epilepsy, vascular conditions, and so on [34]. Medical image analysis is evolving day by day with the development of technology. This is further assisted by 3D virtual model creation as well to improve understanding of complex anatomy and to provide powerful tools for surgical planning and intraoperative guidance. Nowadays, the use of 3D ultrasound and fetal MRI is also becoming common in clinical practice [35]. The interesting fact is how machine learning could be integrated with these medical imaging techniques to make better decisions in surgical planning. It is to be noted that using machine learning, it is possible to understand hidden relationships which may not directly be visible to humans when observing multiple data. This is the reason that even disease predictions in healthcare have been made possible through machine learning approaches. Therefore, by processing these medical image data using unsupervised machine learning techniques such as clustering, an analysis could be performed on the dataset which could later be referred by the surgeon to identify if any crucial information has been lost while planning the surgery or else to even confirm that the decisions made on the approach of conducting the surgery is suitable for the considered patient.

Entities such as lesions and organs in medical images are too complicated and they cannot be shown correctly with the use of simple mathematic solutions. The pixel analysis in machine learning is used for medical image processing from which certain values can be extracted directly from the image. Feature calculation and segmentation is not required in pixel-based machine learning. Due to this, even an image with low contrast will have no issue in processing to extract information. Pixel analysis utilizes longer training time because of the high dimensionality of data. Histogram equalization (HE) is an efficient technique which could be used for contrast improvement. There are various other extensions of HE which were implemented in order to improve the performance of the algorithm. Linear discriminant analysis (LDA), SVM, and DT are few machine learning methods used to analyse medical images. Low binary pattern descriptors are being implemented using machine learning approaches which could be used on biological images. The neural network technique is used in medical images to investigate the details regarding a disease. Machine learning in medical imaging can also be found in medical-based expert systems [16].

The article "Involvement of Machine Learning Tools in Healthcare Decision Making" was published in 2021. Journal: J Healthc Eng.

CNN is one of the best models for image analysis. It has several layers that could convert the input by using convolution filters. There are two sections in classification with regard to medical images. They are image classification and object classification. In image classification, deep learning is used to investigate clinical-related issues so that early treatment for the patient will be possible. In object classification, the main target is to analyse more on interested small chucks of the medical image. In medical image analysis, deep learning algorithms help in categorizing, classifying, and enumerating disease patterns using image processing [16].

Computers have the ability of performing tasks consistently and tirelessly. In the past years, machine learning has proved its ability to learn and master tasks which were considered as too complex for machines to handle, and in some instances, they have been able to identify patterns which are beyond human perception. When using machine learning on medical images, there are few terms which are widely used which need to be discussed. Classification means labelling or assigning a class to a group of pixels. Model is a set of decision points which are learnt by the machine learning algorithm. Algorithm is the steps which have been taken to implement the model. Labelled data are the set of data which are examples for a specific class. Validation set or the training set is the set of data which is used to train the system. Node is a part of a neural network which includes two or more inputs and an activation function. A layer is a combination of nodes from which the outputs are computed. Segmentation is a process of splitting the image into sections so that more focus could be given to the split segments. Overfitting is when a classifier is too specific to the training set and it is not useful as it is only familiar with those examples. Having many features can lead to overfitting. Features are the numeric values that represent the example. When it is with regard to medical images, it can be actual pixel values, edge strengths, variation in pixel values in a region, etc. Feature selection must be done in a way that the selected subset of features is able to provide the best and the most accurate predictions [8].

The article "Involvement of Machine Learning Tools in Healthcare Decision Making" was published in 2021. Journal: J Healthc Eng.

Image recognition and biomedical time series classification are nonlinear classification problems. With the existing classification algorithms and feature extraction technologies, it is not possible to have highly complicated nonlinear functions. But using DNN, nonlinear functions can be constructed by increasing the number of layers and neurons in the network. With the use of ensemble learning, multiple classifiers could also be combined to have complicated decision-making functions. Both in SVM and ensemble learning, nonlinear functions are constructed by combining multiple kernel functions. In the present context, the generation strategy is to later use the same learning algorithm. Therefore, different settings such as learning parameters and training samples are needed. Many methods have been developed having this idea, and they can be divided into four categories. First is to manipulate the training samples. Bagging, boosting, cross-validated committees, wagging, and arcing sort of approaches are needed for this. The second way is to manipulate the input features. Methods such as random subspace, input decimation, and similarity-based feature space can be used for this purpose. The third way is to manipulate the class labels. Output coding and class switching are examples for this. The fourth way is inserting randomness to the learning algorithm. Backpropagation algorithm, randomized first-order inductive learner, and RF are few approaches used for this. The resulting classifiers using backpropagation will be quite diverse if different initial weights are applied to the same training samples in a neural network. Basically, it is visible that the underlying core of the generation strategy is to make the individual classifiers different so that it could be used to improve the classifier performance [36].

## 5. Machine Learning in Biomedicine

Gene expression datasets contain measurements of increasing and decreasing expression levels of a set of genes. Gene expression measurements are usually taken across time points from tissue samples or patients, and they are represented as a matrix of numerical values. In a protein-protein interaction network, the nodes represent biomolecules and the edges represent interactions. In any clustering algorithm, it is always better to have a minimum number of user inputs as it is hard for the users to specify correct values. These user inputs could affect the accuracy of the algorithm if they are incorrect [15].

The article "Involvement of Machine Learning Tools in Healthcare Decision Making" was published in 2021. Journal: J Healthc Eng.

Nowadays, machine learning has become ubiquitous and indispensable when it comes to solving complex problems in many areas. In biomedicine, machine learning is used for various tasks such as to predict protein structure, function from genetic sequences, discern optimal diets from patients clinical and microbiome profile, and so on. Machine learning is also used in processing real-time, high-resolution physiological data in various medical applications. The involvement of machine learning in biomedicine can be discussed mainly in three approaches. First is that machine learning improves prognosis. Current prognostic models are restricted to few variables that humans must enter and tally scores. But these data could be directly taken from EHRs and then it would allow models to use thousands of rich predictor variables which would increase the accuracy of the predictions. Second is that machine learning will reduce the work of radiologists and anatomical pathologists. Normally, these physicians focus on interpreting digitalized images. But using machine learning algorithms, these images can be given as an input, which would result in interpretations and predictions provided by the algorithm. Sometimes, these interpretations even exceed the accuracy of humans. Apart from it, the algorithms do not need rest, and they could work continuously at the same accuracy which is not possible for humans in practice. Third is that machine learning will improve the diagnostic accuracy by minimizing the diagnostic errors. But the challenge which needs to be faced here is the complexity of training the algorithm as the predictions are not binary. Even when working with EHR data, first the data need to be preprocessed to be accessible to the algorithms as they are often stored in an unstructured format.

Data themselves are not useful, but they need to be analysed, interpreted, and acted on to make them useful. Algorithms are required to perform the aforementioned tasks with datasets. Therefore, new statistical tools from the machine learning field are critical when practicing medicine in the present time. Most of the computer-based algorithms in medicine are expert systems. They have a set of rules and knowledge which are being applied to make conclusions with regard to specific clinical scenarios. This is an approach that is similar to a medical student where the general principles about medicine are being applied on new patients. But machine learning is much different than the above discussed, as in a machine learning approach, rules are being learnt from the data themselves. It starts with the patient level observations and checks through vast number of variables to look for combinations that could reliably predict the outcome. The highlight in machine learning is the enormous number of predictors that it handles. Sometimes, there are more predictors than observations and they need to be combined in a nonlinear and highly interactive way to generate accurate outcomes.

The article "Involvement of Machine Learning Tools in Healthcare Decision Making" was published in 2021. Journal: J Healthc Eng.

Truly independent validation datasets must be used from different populations and periods which have no relation with the model development when testing the models. If not in the validation stage, the algorithm will have poor performance. Machine learning algorithms need high-quality data in high quantities to reach acceptable performance levels. If the dataset is biased, it can affect the performance and the generalizability of the algorithm. Machine learning is not capable of solving any fundamental problems of causal inference in the observational dataset. Even though the algorithm is good in predicting the outcomes, yet it is to be noted that these predictors are not the causes [37].

Many research studies have given binary interpretations on whether a person is being diagnosed with a particular disease or not. Sometimes, regarding a particular disease, it may show the stage of the disease as well. It could be noticed that these research studies have been based on a particular disease, but not many diseases together. To address the said limitation, a method was proposed called ensemble label power-set pruned dataset joint decomposition (ELPPJD). The label power-set (LP) method overcomes the independence problem and takes the correlation among labels into consideration. But the issues are that the time complexity increases with the size of the label set and the imbalanced problem keeps on rising when new label sets are produced. Pruned datasets and joint decomposition can be used to overcome these issues. In this approach, when creating new classes, all these training data will be broken down into subsets which are disjoint. Then, using a similarity threshold, the labels which are more similar to each other will be grouped. The subset partition strategies can be size balanced (SB) and label similarity (LS). Random K-label sets (RAKEL) and hierarchy of multilabel classifiers (HOMER) are multilabel classifying methods which can be used as alternatives for this approach. RAKEL runs based on MEKA, and C4.5 is the basic classification algorithm. HOMER runs based on MULAN, and RF is the basic classification algorithm. RAKEL shows better performance than HOMER. But ELPPJD with LS partition strategy outperforms both RAKEL and HOMER [38].

The article "Involvement of Machine Learning Tools in Healthcare Decision Making" was published in 2021. Journal: J Healthc Eng.

## 6. Machine Learning in Biomedical Event Extraction

The relationship between the disease and the drug, the relationship between the disease and the gene, the interaction between drugs, and the interaction between proteins are biological events which have complex structures. To extract these biomedical events accurately and efficiently, biomedical text mining technology is important as the amount of unstructured and semistructured biomedical literature data is rapidly growing.

Pattern-based methods are used in biomedical relation extraction. But they are not much used in biomedical event extraction. Event extraction systems are mainly divided into two types which are rule-based event extraction systems and machine learning-based event extraction systems. In the machine learning approach, the task of extracting biomedical events is considered as a classification problem. The highly unbalanced training dataset given in biomedical event extraction is an issue, and most of the systems do not address this problem. But SVM addresses this issue using the simple class weighting strategy. Machine learning-based event extraction systems have three types. First type is the pipeline model. The pipeline model has achieved excellent results in the event extraction task. But the drawbacks in it are that the time complexity is high and each step is based on the previous step. Therefore, if there is an error, that error would be carried till the final step. Second type is the joint model. This model overcame the previous drawbacks discussed, yet it involves complicated calculations. Third type is the pairwise model. This is a combination of both pipeline and joint models. Pairwise model is faster than the joint model and more accurate than the pipeline model. This model uses SVM to overcome the multiclass and multilabel classification problem without dealing with data imbalance.

A system proposed to extract biomedical events from imbalanced data has several steps. First, text preprocessing will be carried out using token features, sentence features, sentence dependency features, and external resource features. Next is the sample selection, based on sequential patterns. It aims to find the frequent subsequence or sequential events that satisfy the minimum support. This includes the extraction of sequential patterns in the text. Then, the detection of multiargument events is performed, followed by the joint scoring mechanism. This will result in obtaining the outcome. The tool sentence2vec, based on convolutional deep structured semantic models (C-DSSMs), is used to calculate the semantic relevance score [39].

Using SVM, it is possible to separate event extraction into multiple classification tasks, individually detecting the trigger words defining events and the arguments that describe which proteins or genes take part in these events. This is based on labelled data and supervised learning algorithms. But the issue is that these systems get affected by data sparseness. Especially, it happens when the training dataset is too small to find enough information to assign proper weights to those low-frequency or out-of-vocabulary features. Therefore, research was carried out to implement systems that would use the semisupervised or the unsupervised machine learning approach to extract biomedical events. In PubMed, a large pool of unlabelled data with potential information with regard to the biomedical event extraction domain can be found to go ahead with the research. The basic features are obtained by the labelled data and the information which is lacking in labelled data can be obtained from unlabelled data using the event feature coupling generalization strategy. Sparse features that were filtered by supervised machine learning methods can be used to increase the performance of the system while these could even be considered when using a semisupervised machine learning approach for biomedical event extraction [40].

The article "Involvement of Machine Learning Tools in Healthcare Decision Making" was published in 2021. Journal: J Healthc Eng.

Proteins are the end products of a gene expression. Understanding the gene function at the proteome level is a significant interest in the biological and medical research community. There are large repositories of protein data whose characteristics are unknown as noting their functional features using experimental methods have lagged far behind. This creates a need of a computational method to address the issue by accurately working on the large datasets even with a limited amount of labelled data. Functional, structural, and evolutionary characteristics of the protein can be extracted by using the protein sequence information. The aim of protein classification is to extract this information accurately, and it has only been possible with the application of machine learning algorithms to analyse the protein data repositories [41].

## 7. Machine Learning Approaches to Polypharmacology

Polypharmacology focuses on designing medical treatment that can target multiple receptors. The efficacy and toxicity of drugs result from complex interactions between pharmacodynamic, pharmacokinetic, genetic, epigenetic, and environmental factors even though it may be designed as a single or multitarget treatment. Machine learning-related computational techniques are required to enable the prediction and analysis of in vitro and in vivo drug-response phenotypes.

Identification of drug-target interaction on a proteome-wide scale is essential to define and predict a drug response. Apart from its genetic and epigenetic variations, cell-to-cell communication, cell-to-cell variability, and other environmental factors must also be considered. System-based approaches help in drug discovery as they could identify cellular connectivity between all the aforementioned components. New computational methods are needed to accurately calculate free-energy landscapes during association and dissociation of protein-ligand complexes. It will allow to investigate quantitatively both low and high affinity binding on a proteome-wide scale. Self-organizing map is an unsupervised machine learning technique that is used to cluster drug molecules. Prediction of drug-target interactions can be done by combining the sequence features of the receptor with the fingerprint of the ligand, in order to train modules based on statistical machine learning. There are four computational areas which are crucial in polypharmacology, and they are the proteome-wide prediction of drug-target interactions, the quantitative modelling of protein-ligand interactions, the integrated analysis of biological networks, and the dynamic and stoichiometric simulation of biological networks [42].

The article "Involvement of Machine Learning Tools in Healthcare Decision Making" was published in 2021. Journal: J Healthc Eng.

NGS includes both DNA and RNA sequencing. It involves the task of braking DNA and RNA into fragments and determining the order of the nucleotide bases in each fragment. DNA sequencing can either be whole genome sequencing (WGS) or whole exome sequencing (WES) of the coding regions of all known genes and targeted sequencing of genomic regions or genes implicated in a disease. WGS and WES can be found in clinical practices to evaluate developmental brain disorders such as autism, seizures, and intellectual disability. There are commercially available sequencing platforms which use various methods to generate sequence data. With the continuous modifications resulted from the advancement of technologies, NGS-based platforms have shown a comparatively low error rate. In NGS technologies, Sanger sequencing is considered to be the most accurate sequencing method and it is often used for the validation of genetic variants due to its high accuracy [43].

When modern machine learning is combined with medical practice by using clinical data sources, various prediction models could be generated for similar clinical questions. From early warning systems till superhuman imaging diagnostics, there are many applications of machine learning in medical practice. Machine learning methods provide predictions based on existing data. The Google flu reminds how forecasting an annual event based on 1 year of data could lead to time series problems. Having loads of data over the past time has diminishing returns. Basically, it is found in research on decision support algorithms that it is better to use the most recent year data instead of historical data of multiple years for better accurate decisions. Even when evaluating prediction models, the main idea behind this is not about the ability to do repetitions of historical trends but the accuracy it has on predicting future trends. It is true that machine learning algorithms can improve the prediction accuracy by using conventional regression models by capturing complex and nonlinear relationships in the data. But it is to be noted that even though highest computing power is provided, there is no possibility of getting information that is not present. Therefore, using clinical data alone has limited the prediction power. By incorporating the correct data streams, the level of prediction accuracy can be improved. But not even a simple nonlinear system can precisely predict the distant future. Tiny variations which seem nothing and very less important rounding errors can accumulate and make a massive impact on future events [44].

The article "Involvement of Machine Learning Tools in Healthcare Decision Making" was published in 2021. Journal: J Healthc Eng.

## 8. Machine Learning for Drug Repurposing Using System Biology

More than 90% of the drugs that go through the early phases of clinical trials fail due to reasons such as adverse reactions, side effects, or lack of efficiency. To overcome these challenges, drug repurposing has been considered. Repurposing drugs can be either drug-based or disease-based. Drugs that are strongly anticorrelated with a disease are likely to be candidates for repurposing. The connectivity map was the first project that aimed to explore the functional connectivity between drugs. It even considered the functional connectivity between drugs and diseases. Systems biology can be used to discover and develop drugs by giving concern to the interactions of the components in biological entities. Drugs are being ranked based on the amount of perturbation they cause on specific disease-related genes.

A drug disease network (DDN) is constructed by integrating the knowledge on disease-related genes, drug targets, signalling pathways, and gene-gene interactions. The DDN represents all the interactions between drug targets and genes, related to a given disease as described in Kyoto Encyclopaedia of Genes and Genomes (KEGG) signalling pathways. The repurposing scores of the drug-disease pairs are calculated using the Pearson correlation coefficient between their gene perturbation signatures, and it can take a value between 1 to −1. A high positive value indicates that the drug and the disease both cause similar perturbations to the system, and a high negative value indicates that the drug and the disease have opposite gene perturbation signatures. By using this value, it can be recognized whether it is a drug that could be considered as a treatment to a given disease [45].

The article "Involvement of Machine Learning Tools in Healthcare Decision Making" was published in 2021. Journal: J Healthc Eng.

Therefore, it is clear that when a patient approaches and expects support from healthcare, the decision making starts in the process of the patient being diagnosed with a disease and it continues till the proper treatment or medication is prescribed for the patient. In this process, which is a chain of decisions, to support each decision, machine learning approaches are involved in healthcare. Tasks such as predicting or diagnosing a disease, identifying hidden diseases, providing clinical decision support, and even recognizing whether a drug is suitable as a treatment to the given disease are being conducted using machine learning approaches to support clinicians to make fast and accurate decisions. Stepping further ahead, even after a patient is cured from a disease, using machine learning approaches, the EHRs of patients are processed and analysed to identify any future health risks that could possibly occur.

## 9. Discussion

In this section, the main concern would be given towards highlighting important and crucial facts of the topics discussed throughout the paper. To start with, it is better to give concern towards the performance of machine learning algorithms. To identify best performing algorithms, classifier accuracy and the classifier log loss are two factors that can be considered. The classifier accuracy needs to be high and the classifier log loss needs to be low for an algorithm to be identified as a well-performing algorithm. Therefore, once selecting a suitable algorithm to address a specific concern, the aforementioned factors are considered to select the algorithm out of many different existing algorithms that would best suit our purpose.

In most clustering algorithms, the effectiveness of the algorithm depends on the appropriate parameters that the user inputs. For example, parameters like number of expected clusters, a starting point in the dataset, minimum number of samples to form a cluster, and so on affect the clustering result. This is a serious issue when biological and biomedical data are considered as they are nonspherical and high-dimensional. Automatic density clustering method with multiple kernels (ADCMK) is a proposed option to answer the said issue. Using that method, clusters with arbitrary shape can be easily identified based on their density. When comparing the conventional clustering algorithms, ADCMK automatically determines optimal values for the cutoff distance, kernel weights, and number of clusters and centroids which will not change the clustering result when executed time to time. It also has comparatively better accuracy. Multiple kernel clustering approaches help in optimally combining the learning algorithms in order to obtain excellent clustering results and performance in various scenarios. They are mostly suitable to handle labelled datasets as they are a part of supervised kernel learning. There is also an unsupervised multiple kernel learning approach that aims to determine the linear combination of multiple kernels based on an unlabelled dataset [46].

The article "Involvement of Machine Learning Tools in Healthcare Decision Making" was published in 2021. Journal: J Healthc Eng.

It is not possible to exactly highlight which algorithm is better than the other. The reason is that it depends on the domain that the training and the tests are being executed, the dataset that is involved in the training and testing procedures, the level of preprocessing that is being performed on the dataset, the selected feature set for the algorithm or the feature selection algorithms that have been used on the dataset, the size of the dataset and the data types in the dataset, the performance level and the capacity of the machine, and much more. This makes it vital to select the proper algorithm that would be ideal for the requirement. Normally, this cannot be directly selected, but it will be an iterative process to select the most suitable algorithm from a filtered set of algorithms which would best fit the problem in hand. The proper knowledge and past experiences gathered will help in constructing the filtered set of algorithms. When looking at a simple example from the biomedical field, it can be seen that for the diagnosis of various diseases, the best performing algorithm changes due to the aforementioned reason. This could be further explained by looking at the scenarios below, in detail.

Many studies have been carried out using ANN, DT, and LR to diagnose kidney diseases, and ANN has outperformed both DT and LR by a huge margin [26]. According to previous studies, it is to be noted that the accuracy of the results obtained with regard to lung cancer diagnosis is in the order of SVM, ANN, and DT. Apart from them, various other techniques also have been used and they have also showed a reasonable level of accuracy. These algorithms are GA, BPNN, Hopfield neural network, and LDA [30]. Another benefit that could be gained by using SVM classification is that through SVM, it is possible to calculate even the stage of the lung cancer [18]. Regression can be used to model and predict the association between the dependent variable and the independent variable. Regression can be categorized as linear regression and logistic regression. For linear regression, the dependent variable should be continuous, and for logistic regression, the dependent variable should be discrete. Using the logistic regression algorithm to predict complex disease such as cancer must be avoided. KNN is not suitable for cancer predictions as the datasets are huge and more complex which could make the clustering process more difficult [47]. It was found that DNN has better performance for breast cancer detection. Then ANN, SVM, and KNN were ranked in the given order with regard to their performance [48]. It is to be noted that DNN has also shown higher accuracy in predicting diabetics compared with the other standard machine learning algorithms. When discussing extracting of medical data from documents, datasets, databases, medical images, etc. for analysing purposes, various CNN algorithms can be used to extract features from unstructured data. For structured data, NB, KNN, and DT algorithms can be used. For textual data which are unstructured, CNN-based unimodal disease risk prediction (CNN-UDRP) can be used. For both structured and unstructured data, CNN-based multimodal disease risk prediction (CNN-MDRP) can be used. In the CNN-UDRP algorithm, tests are represented in the form of a vector. For each word, the distributed representation of the word embedding found in NLP is used. When working with CNN, it is required to specify the number of words for the sliding window. When assigning a value for the sliding window, it is important to assign a value that would help in reaching the highest accuracy when it is being used [8]. When giving concern to these aspects, what could be seen is how these machine learning approaches assist in healthcare decision making of the clinicians. When analysing reports and when going through the patients' medical history, these algorithms are used to highlight the factors that definitely need to be considered by the clinician when prescribing treatment. In addition to it, these algorithms are also used to assist in identifying the level that the disease has spread in the patient so that the treatment can be given accordingly based on the disease severity.

The article "Involvement of Machine Learning Tools in Healthcare Decision Making" was published in 2021. Journal: J Healthc Eng.

Moving on to the next topic, which is medical imaging, it is visible that currently, medical image classification is mostly based on pattern recognition methods. It has been found that classification-based neural networks have better performance than other supervised machine learning algorithms. Deep learning is considered as a combination of both supervised and unsupervised methods. The reason is that it initially relies on unsupervised learning for training the DNN and then to fine tune the neural network, it uses supervised learning. When compared with various classification algorithms, CNN combined with adaptive sliding window fusion mechanism has good stability and robustness along with high classification accuracy. Even when it is for breast tumour or brain tumour diagnosis, the aforementioned approach with CNN has given comparatively better results [49]. As both deep learning and ensemble learning can construct complicated nonlinear functions, by combining them, it is possible to handle more complex tasks. Biomedical time series often has interfering noise. But when trying to eliminate the noise, along with it some useful information might also be lost. DNN has the ability to capture useful information while ignoring the interfering noise after learning from training samples. Presently, DNN mainly includes CNN, deep belief network (DBN), and autoencoder (AE). CNN performs convolution operations on both horizontal and vertical directions. This is a good approach for image data as it is relevant in both directions. But for biomedical time series with multiple channels, this is not suitable as only horizontal direction is relevant and the vertical direction is independent. For this reason, multichannel CNN can also be implemented to obtain better classification performance [36].

When further observed, it is also visible that in the present context, medical imaging has also been combined with the 3D printing technology to achieve greater success specially when surgical planning is to be considered. 3D printing can turn a 3D medical image dataset into a 3D object as per the patient's actual size. This can largely improve the precision of modern surgical planning by combining with other preoperative plan and intraoperative navigation techniques. By combining these with the cloud computing architecture, there is further space for improvement in cost efficiency, flexibility, and clinical workflow. Therefore, further exploration needs to be done on 3D printing and cloud computing technologies of their usage in the surgical realm. Nowadays, surgeons are able to perform risky procedures with high level of safety and accuracy with the development of multimodality imaging, with regard to especially the fusion of functional imaging in preoperative planning and modern image guided therapy in intraoperative navigation. With the development of medical imaging technology, there are multiple imaging processing systems and intraoperative imaging guided platforms which are being introduced that are powerful but also complicated [50]. In addition to it, 3D printing has also been used to design advanced prosthetic devices with the aim of developing a realistic model which is closely similar to the actual part with regard to the geometry and mechanical properties. When making such products, even though the geometry can be easily obtained by the 3D scanned data, the mechanical properties need to be mechanically validated and a major concern should be given towards composite material technology [51]. A few of the currently existing findings on prosthetic devices are briefly discussed below.

The article "Involvement of Machine Learning Tools in Healthcare Decision Making" was published in 2021. Journal: J Healthc Eng.

The concept of creating a soft total artificial heart from silicon elastomers using the lost-wax casting technique has also been possible as the 3D printing technology has enabled the production of entirely soft pumps with complex chamber geometries. Even though it is not yet readily implantable, it promotes the future of personalized medicine and artificial heart development without requiring expensive and complex equipment [52]. By using an array of semiconductor photo detectors which are made of polymers and printed on a glass hemisphere, a 3D printed prototype of a bionic eye has been designed and further research is being carried out on ways to improve the efficiency of the photo detectors and to find a way to print on a soft hemispherical material that could be implanted to a real human eye [53]. Researchers have also developed a 3D printed tooth that also kills bacteria using conventional artificial tooth resins combined with positively charged quaternary ammonium ions [54]. In another study, a handheld portable printer was developed which could be used to create narrow sheets of skin tissue made from collagen and fibrin to cover and heal deep wounds. This printer can tailor tissues based on the patient and the wound characteristics within two minutes or less. Further research is being carried out on ways to expand the size of the printed strips so that larger wounds could be covered [55]. Bioengineers have 3D printed artificial hyperelastic bones which could quickly induce bone regeneration and growth. Currently, it has been implanted successfully in animal models and a main advantage in this approach is that the 3D printing process can customize any shape of a bone as per the requirement and can create it within a day. It is to be noted that the materials used to create these 3D printed bones are flexible, and after combining them with the bone structure, with time, they bond with the existing bones and become a part of the human body [56]. A group of scientists has 3D printed a bionic ear with an antenna and a cartilage that can hear the radio frequencies even beyond the range of a normal human's capability. It has also been created in such a way that the electrical signals produced from the ear can be connected with the nerve endings which is considered to be the first time that 3D printing was effectively used to interweave tissues with electronics [57]. There are many such prosthetic devices which were outcomes of previous research studies that were carried out, and further research is being conducted on them presently to improve the existing results. Medical imaging, 3D printing technologies, and various other computational approaches have been vital when conducting these research studies to obtain improved results. When giving concern to how machine learning could be involved in these findings, it is visible that machine learning approaches could analyse large biological and material datasets to identify various relationships which exist between the data. In addition to it, as machine learning is used to detect diseases and the severity level of it, these machine learning algorithms can be combined with the equipment that is being used to design such prosthetic devices so that when the medical dataset is given, an analysis is to be performed so that the devices can be customized and designed based on the patient's requirement which would further encourage the latest trend in healthcare, which is personalized medicine.

The article "Involvement of Machine Learning Tools in Healthcare Decision Making" was published in 2021. Journal: J Healthc Eng.

When discussing biomedicine, biomedical data play an important role which cannot be neglected. It is vital to extract the required knowledge from biomedical data that would make paths visible to explore the subject matters further. When giving concern towards bioinformatics and biomedical data, there are various documents that contain high-dimensional data with large number of attributes such as categorical images and text records. To extract information from such documents efficiently and with high accuracy, t-distributed stochastic neighbour embedding method could be used. It is a popular method for exploring high-dimensional data in the field of machine learning and can be incorporated with the multiple kernel approach as well. ADCMK performs data preprocessing, optimal combined kernel determination, cluster centroid detection, and assignment and visualization of clusters which shows excellent results when working with larger-scale biological and biomedical datasets without class label information [46].

Under biomedical event extraction, the challenges that protein classification tasks need to face due to the limited data that are available for learning and the unbalanced classes in those existing data need to be considered and addressed. Expectation-maximization-based algorithms are there to address these challenges by incorporating unlabelled data. Even by using the n-gram model for the feature space with the NB classifier, the accuracy of the model could be improved to some extent without using unlabelled data. The transductive support vector machine (TSVM) method is a semisupervised learning approach that also could be used in addressing the said issues. But there are other semisupervised algorithms as well that could perform better in certain classification problems [41].

The article "Involvement of Machine Learning Tools in Healthcare Decision Making" was published in 2021. Journal: J Healthc Eng.

While coming towards the machine learning approaches to polypharmacology, it is important to recognize about certain risks or loopholes which can be found when integrating machine learning algorithms with biology and biomedicine. In some occasions, there may be identical twins with the same observable demographic characteristics, lifestyle, medical care, and genetics which will provide same predictions by a machine learning algorithm but will end up in totally unexpected different outcomes. This is an instance to show that the incorporation of machine learning with biology and biomedicine should be performed with maximum care and monitoring. Research studies are growing in number trying to increase the accuracy of the predictions made, but still these algorithms do not state how to change the obtained outcome. It even does not assure whether it is possible to change the received outcomes in any possible way. Machine learning-based identifications are strong, but they are theory free. This means that no theory-based explanations can be provided, even for the generated predictions. Sometimes, the most accurate predictions made by machine learning algorithms are obvious to the practicing clinicians as well. Even though predictive algorithms cannot eliminate medical uncertainty, they improve allocation of scarce healthcare resources. Using DNN, now early warning systems can be rapidly developed and optimized using real-world data. These systems will also have capabilities which seemed to be impossible to be achieved previously [44].

Here onwards the discussion will give concern towards increasing the productivity of applications through increasing the performance of the machine learning algorithms. In order to increase the performance and the efficiency of machine learning algorithms, various steps and measures are being carried out and tested by the researchers. When observing the said fact, next are a few instances to get an idea of what sort of tasks are being conducted to increase the performance of the algorithms. When considering the accuracy, sensitivity, and the specificity of classifiers while changing the number of folds, any major fluctuation was not found in the values obtained in the confusion matrix. All were just small variations in the final decimal places which can be ignored [26]. But DNN, feature selection methods, and cross validation techniques can be applied to increase the classification accuracy [10, 58]. It is also to be noted that positive predictive value (PPV), negative predictive value (NPV), accuracy, sensitivity, and specificity attributes show an improvement when a classifier is applied after performing PCA rather than the classifier being applied to the official feature set (OFS). But when the GA was used instead of the PCA, all the above attributes showed a further improvement even than what was resulted after the PCA has been applied [29].

The article "Involvement of Machine Learning Tools in Healthcare Decision Making" was published in 2021. Journal: J Healthc Eng.

Ensemble learner is constructed by a collection of individual classifiers. When there is a pattern classification problem, it is solved by a combination of multiple classifier outputs. Majority voting, bagging, and boosting are few well-known ensemble methods which can be used to combine the outputs. Normally, this approach is more accurate than using a single classifier. In the majority voting method, the label to be assigned is decided based on the majority of the individual classifier's outputs. The bagging method decreases the variance of the predictions by generating additional data for training from the original dataset. The boosting method has two steps. The first is using the original data to produce a series of averagely performing models. Then, the next step is to increase the performance by combining the previous performances using a voting scheme [10]. Using the ensemble technique, a weak classifier can be converted to a strong classifier. When working with a weak classifier, it is merged using the weighted average of the prediction accuracy as metrics. Then, the error will be propagated with every prediction, and until the prediction becomes accurate, multiple iterations will be carried out to reduce the error [59].

Maximum sensitivity neural networks use the backpropagation algorithm to adjust the weights associated with the neurons. This is special as it saves time and memory while predicting more accurately as the output layer detects the maximum sensitivity of the neurons for the new pattern [47].

Machine learning feature extraction is the process that helps in identifying the relevant attributes from various candidate subnets, and it plays a vital role in creating an effective predictive model. There are various benefits of applying feature selection, such as highly effective and fast training of the machine learning algorithm, reducing the complexity of the model, improving the accuracy of the model, and eliminating the overfitting problem. There are three groups that could be identified in feature selection methods. They are filter, wrapper, and embedded methods. The filter method is normally a preprocessing step that relies on general features. The wrapper method uses machine learning in order to select the best and the most suited subset of features. Forward feature selection, backward feature elimination, and recursive feature elimination are widely used wrapper methods. The embedded method combines the qualities of the filter and wrapper methods [17]. It is important to remember that when features are correlated to other features, there is no point having all of them considered in the machine learning algorithm as it will increase only the execution time but will not improve the efficiency of the algorithm. It is also to be noted that when adding certain features, the accuracy of the algorithm may drop. It is preferred if each of the features could be tested individually and then combined in a way that the accuracy of the output will be increased [27]. The quality of the feature selection process has a direct impact on the accuracy increase. Some algorithms like ANN show a higher increase in the accuracy when compared with other algorithms after the feature selection phase is performed [25].

The article "Involvement of Machine Learning Tools in Healthcare Decision Making" was published in 2021. Journal: J Healthc Eng.

Machine learning techniques have gained significantly high accuracy when considering classification-based problems. A four-tier architecture can be used to store and process a huge volume of data efficiently. Tier 1 can be used to collect data, and tier 2 can be used to store huge volumes of data. Tier 3 and tier 4 can be used for machine learning classifications and representation of the results, respectively [14]. In the present time, as computing power is not an issue, DNN has more than 20 layers. Early neural networks were typically less than 5 layers. DNNs are used for various purposes such as automatic object detection, segmentation on images, automatic speech recognition, genotypic and phenotypic detection, classification of diseases in bioinformatics, and so on. Even though CNN is quite similar to regular neural networks, it assumes that there are geometric relationships among inputs. By using convolutional layers in DNN, important features could be amplified for better analysis. The pooling layer in CNN takes the output and finds the maximal value so that it could give the convolution function the best extracts of the images. Regularization is used when training deep networks as it increases the performance by reducing overfitting. There are no exact number of layers to obtain more accurate results, but it is an iterative trial and error process in which the best architecture needs to be found for a specific problem. The advantage of using CNN over traditional machine learning algorithms is that there is no need to compute the features as the first step. But CNN will find the important features as a part of its searching process [8].

The article "Involvement of Machine Learning Tools in Healthcare Decision Making" was published in 2021. Journal: J Healthc Eng.

As ANN is complex, other simple machine learning algorithms such as SVM, KNN, and RF gradually came ahead of ANN in popularity. By selecting the appropriate activation functions, better feature extraction can be achieved, as they are what form the nonlinear layers in deep learning frameworks. There are many activation functions. Sigmoid function, hyperbolic tangent, softmax, rectified linear unit (ReLU), softplus, absolute value rectification, and maxout are a few of such commonly used activation functions. There are various deep learning architectures such as AE, DBN, restricted Boltzmann machines (RBM), CNN, and RNN. AE is different from ordinary ANN as it extracts features from unlabelled data and sets target values to be equal to the inputs. RBMs are generative graphical models and their aim is to learn the distribution of the training data. DBM can be considered as a stack of AEs or RBMs. CNN is different from other deep learning algorithms as it extracts features from small sections of an input image. RNN outperforms all the other deep learning approaches when it is about dealing with sequential data. Machine learning is widely used in the medical image domain. Sparse autoencoder (SAE) and RBM can deal with dynamic data and they can also extract patterns from unlabelled data. Due to its capacity of analysing special data, CNN is used in biomedical image analysis commonly. When considering the challenges, it is to note that in deep learning, it requires a large amount of labelled data for model training. Another issue when working with biomedical data is that they are imbalanced, as the normal people set is much larger than the diagnosed people set. They also need high memory and high computing power. The input images must be in high resolution. Nowadays, there are various medical devices and sensors which provide large amounts of data. Deep learning approaches are good interpreters of these data for disease prediction, prevention, and diagnosis.  Table 1 lists few applications of the above-discussed deep learning algorithms in the field of biology and biomedicine [60].

As per Table 2, there are several open-source machine learning libraries in various languages which could be used to assist in the development process when implementing intelligent biological applications. Python and C++ have the most number of libraries that support deep learning. But Python is more often used in traditional machine learning approaches [60]. The popularity or the usage of various deep learning frameworks in projects, when categorized based on the language that they are written in, is shown in Figure 1.

The article "Involvement of Machine Learning Tools in Healthcare Decision Making" was published in 2021. Journal: J Healthc Eng.

At the initial stage, simple machine learning classifying and clustering algorithms were used in data processing and predictions, but when moving forward, with the development in computational power and programming methodologies, more enhanced and complex machine learning algorithms were adapted by the field of biology and biomedicine to obtain more accurate results at a higher efficiency. Even at this very moment various attempts are being executed to further evolve the computational biology and biomedicine domain with the integration of sophisticated scalable machine learning algorithms. Many languages provide multiple application program interfaces (APIs) and libraries in order to assist in these development processes so that the main concern or priority could be given to the requirement with regard to the subject matter and less attention towards the efficiency and performance of the algorithms, as they have already been handled by the libraries or APIs. These algorithms could even be applied to different domains such as marketing, social media, search engines, fraud detection, stock market analysis, e-business, authentication, and so on by changing the training datasets and the features to be analysed. But in this review paper, the computational biology and biomedicine domain was considered.

When coming back to precision medicine, as discussed previously, the simplest definition that could be provided would be treating patients based on their genetic, lifestyle, and environmental data. This is simply not an easy task. It needs to have a whole load of data that should be analysed to obtain the required knowledge for it. This is near impossible for humans to manually process. Furthermore, some relationships among data cannot be identified by humans after exploring the dataset. But as discussed previously, unsupervised machine learning has been able to capture these relationships and group data according to the identified relationships. As precision medicine studies are involved with genes, it is certain that the biomedical event extraction would also contribute towards it. For a patient to then be treated using precision medicine, few approaches in computational biology are vital, such as biomedical data analysis, disease diagnosis, and medical image analysis. The reason is that categorizing the patients to identify the treatment to be followed according to a set of considered factors needs better observations of the patient and his/her medical history.

Throughout this paper, on many occasions, the involvement of machine learning in computational biology and biomedicine has been discussed. The reason behind it is that more than 80% of the healthcare decisions are made based on the said areas. In addition to it, data analytics is being applied in the healthcare sector to improve the healthcare services by predicting the future expectations based on a patient's medical history. Therefore, there is no doubt that prominent attention needs to be given towards the areas of computational biology and biomedicine when discussing computational decision making in healthcare. But it is to be highlighted that whenever we use an approach related to artificial intelligence in healthcare, it is always related to making a decision. Disease detection, disease prediction, drug repurposing, precision medicine, medical resource allocation, and much more can be shown as evidence for it. In all of them, a machine learning algorithm either makes a decision or least it would support a decision. It helps in solving a doubt that a clinician may have or sometimes highlighting a fact which was not visible to the clinician at the time of making a decision as a solution for a healthcare-related issue. In addition to it, most importantly, it deals with people's lives and even a simple mistake can make a huge impact on a person and even the society at large. Therefore, computational decision making is so crucial in the healthcare sector to make confident and accurate decisions in less time and at low cost. This has only been possible with machine learning approaches being adapted as a tool in healthcare and is currently being extensively applied in healthcare decisions.

The article "Involvement of Machine Learning Tools in Healthcare Decision Making" was published in 2021. Journal: J Healthc Eng.

## 10. Conclusion

While reaching the end of the paper, there is no doubt that machine learning algorithms, which is a subsection of artificial intelligence, have inspired the field of computational biology and have contributed immensely to the healthcare sector in terms of fast, efficient, accurate, and cost-effective computational decision making. It is clearly visible that in the present context, machine learning has been applied in various sections in the discussed field. The involvement of machine learning can be found in disease diagnosis and prediction, medical imaging, drug repurposing, biomedical event extraction, and much more in healthcare. But what is certain is that the journey that started with the integration of machine learning to computational biology has come a long way passing several milestones and is now at a peak with the introduction of precision medicine. When considering all the above applications of machine learning in healthcare, what is clearly visible is that how artificial intelligence has been a key resource area for decision making in the healthcare sector in various aspects. When giving concern to the most recent applications of artificial intelligence in healthcare, the best example would be how different tasks such as patient care, treatment research, resource allocations based on the hospital volume, predictions and preparing for future possible requirement, and so on were handled and managed during the COVID-19 pandemic. With all that being said, it is crystal clear that artificial intelligence had played a huge role through machine learning to implement computational decision making tools for the healthcare sector, and in present times, they are of much importance and could not be separated from the healthcare sector.

The article "Involvement of Machine Learning Tools in Healthcare Decision Making" was published in 2021. Journal: J Healthc Eng.

## Figures and Tables

**Figure 1:** Popularity of deep learning frameworks [60].

**Table 1:** Applications of deep learning algorithms in computational biology [60].

Deep learning algorithm	Medical image analysis	Protein structure prediction	Genomic sequencing and gene expression analysis
Convolutional neural network	Brain tumour segmentation, knee cartilage segmentation, prediction of semantic descriptions from medical images, segmentation of MR brain images, coronary artery calcium scoring in CT images	Prediction of protein order/disorder regions, prediction of protein secondary structures, prediction of protein structure properties	—
Sparse autoencoder	Organ detection in 4D patient data, segmentation of hippocampus from infant brains, histological characterization of healthy skin and healing wounds	Sequence-based prediction of backbone C*α* angles and dihedrals	—
Deep belief network	Segmentation of left ventricle of the heart from MR data, discrimination of retinal-based diseases	Prediction of protein disorder, prediction of secondary structures, local backbone angles	Modelling structural binding preferences and predicting binding sites of RNA-binding proteins, prediction of splice junction at DNA level
Deep neural network	Brain tumour segmentation in MR images, prostate MR segmentation, gland instance segmentation	—	Gene expression inference, prediction of enhancer, prediction of splicing patterns in individual tissues and differences in splicing patterns across tissues
Recurrent neural network	Classification of patterns of EEG synchronization for seizure prediction, EEG-based lapse detection	Prediction of protein secondary structure, prediction of protein contact map	Prediction of miRNA precursor and miRNA targets, detection of splice junctions from DNA sequences

**Table 2:** Machine learning libraries in languages [8].

Language	Traditional machine learning libraries	Deep neural network machine learning libraries
Python	Scikit-learn, PyBrain, Nilearn, Pattern, MILK, Mixtend	Keras, Tensorflow (written in both C++ and Python), Nolearn, DeePy, Pylearn2
R	Caret, Boruta, GMMBoost, H2O, KlaR, rminer	Darch, DeepNet
C++	Shogun	Caffe, EBLearn, Intel Deep learning Framework, Tensorflow (written in both C++ and Python)
Java	Encog, Spark, Mahout, MALLET, Weka	Deeplearning4j
JavaScript	Cluster, LDA, Node-SVM	ConvnetJS
